The article "Genistein inhibits stemness of SKOV3 cells induced by macrophages co-cultured with ovarian cancer stem-like cells through IL-8/STAT3 axis" was retracted in 2023. Reasons: duplicated images; original data or images not available; unreliable results or conclusions.

# Genistein inhibits stemness of SKOV3 cells induced by macrophages co-cultured with ovarian cancer stem-like cells through IL-8/STAT3 axis

**DOI:** 10.1186/s13046-018-1010-1

**Published:** 2019-01-15

**Authors:** Yingxia Ning, Weifeng Feng, Xiaocheng Cao, Kaiqun Ren, Meifang Quan, A. Chen, Chang Xu, Yebei Qiu, Jianguo Cao, Xiang Li, Xin Luo

**Affiliations:** 1 Department of Gynaecology and Obstetrics, The First Affiliated Hospital of Guangzhou Medical University, Guangzhou, 510120 China; 2 The First Affiliated Hospital of Jinan University, Guangzhou, 510632 China; 3 Department of preclinical medicine, Medical College, Hunan Normal University, Changsha, 410013 China; 4 Department of Pharmaceutical Science, Medical College, Hunan Normal University, Changsha, 410013 China; 5 Key Laboratory of Study and Discover of Small Targeted Molecules of Hunan Province, Changsha, 410013 China

**Keywords:** Ovarian cancer, Tumor associated macrophages, Ovarian cancer stem-like cells, Genistein, IL-8/STAT3 axis

## Abstract

**Background:**

Recent studies showed that macrophages co-cultured with ovarian cancer stem-like cells (OCSLCs) induced SKOV3 cell stemness via IL-8/STAT3 signaling. Genistein (GEN) demonstrates chemopreventive activity in inflammation-associated cancers. The present study aimed to examine whether and if GEN inhibits the stemness of SKOV3 and OVCA-3R cells induced by co-culture of THP-1 macrophages and SKOV3-derived OCSLCs.

**Methods:**

The co-culture was treated with or without different concentrations (10, 20, and 40 μmol/L) of GEN for 24 h. Depletion or addition of IL-8 in Co-CM and knockdown or overexpression of STAT3 in THP-1 macrophages was performed to demonstrate the possible associated mechanisms. The combined effects of GEN and STAT3 knockdown were examined with the nude mouse modle by co-injection of SKOV3-derived OCSLCs with THP-1 macrophages.

**Results:**

Our results showed that GEN down-regulated CD163 and p-STAT3 expression of THP-1 macrophage, decreased the levels of IL-10, increased the levels of IL-12 and nitric oxide (NO) in the conditioned medium, and reduced the clonogenic and sphere-forming capacities and the expression of CD133 and CD44 in SKOV3 cells induced by co-culture of THP-1 macrophages and OCSLCs in a dose-dependent manner. Moreover, depletion or addition of IL-8 enhanced or attenuated the effect of GEN. Additionally, knockdown or overepression of STAT3 in THP-1 macrophages potentiated or attenuated the inhibitory effects of GEN. Importantly, STAT3 overexpression retrieved the effects of IL-8 combined with GEN depletion on M2 polarization of THP-1 macrophages and stemness of SKOV3 cells induced by co-culture. The combination of GEN and STAT3 knockdown cooperatively inhibited the growth of tumors co-inoculated with OCSLCs/THP-1 macrophages in nude mice in vivo through blocking IL-8/STAT3 signaling.

The article "Genistein inhibits stemness of SKOV3 cells induced by macrophages co-cultured with ovarian cancer stem-like cells through IL-8/STAT3 axis" was retracted in 2023. Reasons: duplicated images; original data or images not available; unreliable results or conclusions.

**Conclusions:**

In summary, our findings suggested that GEN can inhibit the increased M2 polarization of macrophages and stemness of ovarian cancer cells by co-culture of macrophages with OCSLCs through disrupting IL-8/STAT3 signaling axis. This assisted GEN to be as a potential chemotherapeutic agent in human ovarian cancer.

**Electronic supplementary material:**

The online version of this article (10.1186/s13046-018-1010-1) contains supplementary material, which is available to authorized users.

## Background

Ovarian cancer is the most frequently diagnosed tumor and lethal gynecological malignancy in the globe. Owing to the non-specific symptoms associated with the disease, most of the ovarian cancer cases are presented with advanced stage disease and lead to high mortality rates [1, 2]. Despite modest improvements in response rates, progression-free and median survival rates using adjuvant platinum and taxane chemotherapy following cytoreductive surgery, the overall survival rates for patients with advanced ovarian cancer remain disappointing [3, 4]. This is thought to be due to a small subset of cells within the tumor, namely ovarian cancer stem-like cells (OCSLCs) that are resistant to conventional chemotherapy treatments [5]. Current chemotherapy agents aimed on the rapidly dividing cells; however, OCSLCs are not effectively killed by these compounds duo to their slow-division [6, 7]. Therefore, finding and developing a candidate agent that target OCSLCs for the treatment of human ovarian cancer remains important and has clinical implications.

Jackson et al. reported that spheres derived from SKOV3 cells have relatively strong growth potential both in vivo and in vitro compared with the monolayer, indicating that the spheres have the characteristics of OCSLCs [8]. We have recently used stem cell conditioned culture system to obtain the second generation spheres derived from SKOV3 cells, followed by demonstrated the spheres have the characteristics of cancer stem cells (CSCs), considering them as SKOV3-derived OCSLCs [9, 10]. Nowadays, the tumor infiltrating inflammatory cells are mainly considered as tumor associated macrophages (TAMs), which play an important role in tumorigenesis, cancer invasion and metastasis [11, 12]. Recent studies have shown that the interaction of TAM and OCSLCs is involved in the occurrence, recurrence and multidrug resistance of ovarian cancers [13, 14]. Our previous study showed that THP-1 macrophages co-cultured with SKOV3-derived OCSLCs contain the characteristics of TAMs [15]. In this study, we thus used the co-culture of THP-1 macrophages and SKOV3-derived OCSLCs to establish an experimental system for interaction between TAM and OCSLCs.

The article "Genistein inhibits stemness of SKOV3 cells induced by macrophages co-cultured with ovarian cancer stem-like cells through IL-8/STAT3 axis" was retracted in 2023. Reasons: duplicated images; original data or images not available; unreliable results or conclusions.

Importantly, several studies have confirmed that signal transducer and activator of transcription 3 (STAT3) activation is involved in the interaction between CSCs and their microenvironment, which effectively promoted the characterization of CSCs [16–18]. Furthermore, interleukin-8 (IL-8) triggers the activation of STAT3 signaling, which is associated with inflammation, production of reactive oxygen species, ovarian cancer tumorigenesis and multidrug resistance [19, 20]. Mohamed et al reported that IL-8 secreted from macrophages of patients with inflammatory breast cancer is involved in enhancing migration, invasion and metastasis [21]. Tsuyada et al reported that breast cancer cells secrete multiple cytokines and activate STAT3 induced from breast cancer associated fibroblasts [22]. The study conducted in our laboratory showed that OCSLCs co-cultured with macrophages induced SKOV3 cell stemness via IL-8/STAT3 signaling [15]. These data indicated that blocking IL-8/STAT3 signaling of TAMs can evidently hinder the communication between the tumor and the host stromal cells, suggesting it as a novel therapeutic target for cancer stem cells that mediate the evolution of ovarian cancer and other malignant diseases.

Several comparative studies reported that the levels of soy products and isoflavones were negatively correlated with the incidence of various cancers, including ovarian cancer [23–25]. In vitro and in vivo analyses showed that genistein (GEN), an isoflavone compound that is derived from legumes and dentate plants, inhibited oncogenicities in several cancer cells, including cancer stem cell like cells (CSLCs) [26]. GEN has also been reported to display chemopreventive activity in inflammation-associated cancers [27]. Accordingly, we aimed to assess whether and how GEN inhibits the stemness of ovarian cancer cells induced by co-culturing of THP-1 macrophages and OCSLCs.

## Methods

### Cell line and co-culture

Human ovarian cancer SKOV3 and OVCAR-3 cells and human monocyte THP-1 cells were obtained from the cell bank of Chinese Academy of Sciences (Shanghai, China).

SKOV3 and OVCAR-3 cells were cultured in Dulbecco’s modified Eagle’s medium (DMEM) with high glucose (Gibco, Grand Island, NY, USA), containing 10% fetal bovine serum (FBS), 100 IU/ml penicillin, and 100 μg/ml streptomycin, and then were incubated at 37 °C in an atmosphere with 5% CO_2_. The second generation spheres of SKOV3 cells were obtained using sphere-forming assay, and then were considered as OCSLCs [15].

The article "Genistein inhibits stemness of SKOV3 cells induced by macrophages co-cultured with ovarian cancer stem-like cells through IL-8/STAT3 axis" was retracted in 2023. Reasons: duplicated images; original data or images not available; unreliable results or conclusions.

THP-1 cells were cultured in RPMI-1640 medium (Gibco, USA) supplemented with 10% FBS (Gibco, USA), 100 IU/ml penicillin G, and 100 μg/ml streptomycin, and then were incubated in a humidified atmosphere of 5% CO_2_ at 37 °C. THP-1 macrophages were induced by phorbol-12-myristate-13-acetate (PMA; final concentration: 100 ng/ml) for 24 h. Activated THP-1 macrophages were obtained as previously described [15]. In brief, the THP-1 macrophages (2 × 10^6^) were plated in the lower chamber and cultured for 12 h. Then the SKOV3- and OVCAR-3-derived OCSLCs (2 × 10^6^) were seeded in the upper chamber and co-cultured for 24 h in transwell system (BD Biosciences, San Jose, CA, USA). After that, the THP-1 macrophages activated OCSLCs in the lower chamber and the supernatant of co-culture (Co-CM) were collected.

### Spheroid formation assay

SKOV3 and OVCAR-3 cells (2 × 10^3^) were suspended in serum-free DMEM/F12 mixture containing 100 IU/ml penicillin, 100 μg/ml streptomycin, 20 ng/ml hrEGF, 20 ng/ml hbFGF, 0.2% B27, 0.4% BSA, and 4 μg/ml insulin (cancer stem cell conditioned medium, CSC-CM) as well as Co-CM (*v*/v: 1:1). The cells were then seeded in an ultra low attachment 6-well plate (Corning Inc., Coring, NY, USA). The total number of tumor spheres was counted after culturing for 8 days. The efficiency of sphere formation was calculated as previously described [15]. Three independent experiments were performed.

### Colony formation test

DMEM medium containing 0.7% agarose was added into a 6-well plate. Then, 10^4^ SKOV3 and OVACR-3 cells were seeded per well in CSC-CM as well as Co-CM (v/v: 1:1) containing 0.4% agarose (top layer), and incubated for 3 weeks. Colony count was carried out by using an inverted microscope (Olympus IX53, Japan). Three independent experiments were performed.

### Depletion of IL-8 or addition of IL-8

Co-CM was collected, and was incubated with IL-8 neutralizing antibody (50 nM) (PeproTechInc, USA) for overnight at 4 °C. Then the medium was centrifuged at 12,000 g for 10 min, and the supernatants were collected for use as conditioned medium for IL-8 immunodepletion. Collected Co-CM was mixed with sterile 10 ng/ml of recombinant human IL-8 (R&D Systems, USA), and this was considered as the conditioned medium for adding IL-8.

### Adenovirus infection

THP-1 macrophages (1 × 10^5^) were seeded into 6-well culture plates (Corning Inc.) and incubated overnight until they reach 50% confluence, and infected with adenoviral particles loaded with pHBad-MCMV-EGFP-STAT3, pHBad-MCMV-EGFP, pHBad-U6-GFP-shSTAT3, and pHBad-U6-GFP plasmids (Hanbio Biotechnology Co. Ltd., Shanghai, China), respectively. The cells were cultured with Opti-MEM containing 50.0 μL adenoviral particles (Han Heng Biotech Corp) using Enhanced Infection Solution (Jikai gene Co., Ltd., Shanghai, China) for 2 h, and after which, the medium was replaced with DMEM containing 10% FBS. Infection efficiency was calculated by counting GFP-positive cells and live cells using the same high power field under a fluorescent microscope (Olympus IX53, Japan).

The article "Genistein inhibits stemness of SKOV3 cells induced by macrophages co-cultured with ovarian cancer stem-like cells through IL-8/STAT3 axis" was retracted in 2023. Reasons: duplicated images; original data or images not available; unreliable results or conclusions.

### Enzyme-linked immunosorbent assay

Co-CM was collected from SKOV3- or OVCAR-3-derived OCSLC/THP-1 macrophage co-cultures, centrifuged at 1000 g for 5 min to obtain the supernatants, and then assessed for IL-10, IL-12, and IL-8 levels by ELISA with specific kits (Neobioscience, Shenzhen, Guangdong, China) according to the manufacturer’s instructions. Absorbance was immediately read at 450 nm on a microplate reader (BioTek, Winooski, Vermont, USA).

### GEN treatment in vitro

To examine the effects of GEN on co-cultures, THP-1 macrophages co-cultured with SKOV3- or OVCAR-3-derived OCSLCs were treated with or without different concentrations of GEN (10, 20, and 40 μmol/L) for 24 h. For determining the induced effects of GEN combined with depletion or addition of Co-CM on macrophage polarization and SKOV3 cell stemness, the THP-1 macrophages and SKOV3 cells were treated with or without the conditioned medium from Co-CM depleted IL-8 by neutralizing antibody or added recombinant human IL-8 in the presence or absence of GEN (10 μM). To evaluate the linkage between STAT3 activation in THP-1 macrophages and GEN treatment in co-cultured THP-1 macrophages with SKOV3-derived OCSLCs, the co-culture of THP-1 macrophages expressing STAT3 or STAT3 shRNA or both with SKOV3-derived OCSLCs were treated with or without GEN (10 μM).

### Western blot analysis

The cells were harvested and lysed using ice-cold RIPA lysis buffer (Beyotime Biotechnology, CN). Bradford assay (Bio-Rad Laboratories, Hercules, USA) was used to determine the protein concentration. Equal amounts of protein (40 μg) were separated by 10% sodium dodecyl sulfate-polyacrylamide gel electrophoresis (SDS-PAGE), and then transferred onto a polyvinylidenedifluoride membrane (Millipore, Billerica, USA). The membranes were then blocked with TBST supplemented with 5% BSA for 2 h at room temperature, and incubated with primary antibodies against CD133, CD44, CD163 and STAT3 (Abcam, Burlingame, USA, dilution of 1:2000), Nanog and Oct4 (Cell Signaling Technology; Danvers, MA, USA), p-STAT3 (Tyr 705) and β-actin (Santa Cruz, USA, dilution of 1:2000) for overnight at 4 °C. The membranes were incubated with a horseradish peroxidase-conjugated goat anti-mouse IgG antibody or goat anti-rabbit IgG antibody (Beyotime Institute of Biotechnology, Shanghai, China) for 1 h. The protein bands were detected using enhanced chemiluminescence kit (Amersham Biosciences, Piscataway, USA).

The article "Genistein inhibits stemness of SKOV3 cells induced by macrophages co-cultured with ovarian cancer stem-like cells through IL-8/STAT3 axis" was retracted in 2023. Reasons: duplicated images; original data or images not available; unreliable results or conclusions.

### In vivo tumorigenicity experiments

Female BALB/c-nude mice (4–5 weeks of age, body weight 12–14 g) were purchased from Nanjing Institute of Biomedical Research in Nanjing University. The experimental procedure was performed in accordance with the standard protocols and approved by the Ethics Committee of Hunan Normal University (No. 2015–055) and the Committee of Experimental Animal Feeding and Management (ID: 201607119). Mice were acclimated to their new environment for 1 week prior to undergoing the experiment.

To determine that effects of interaction between SKOV3-derived OCSLCs and THP-1 macrophages on the growth of tumors in nude mice in vivo, the mice were injected with SKOV3-derived OCSLCs (1 × 10^5^ cells) in the left flank, and co-injected OCSLCs (1 × 10^5^ cells)/THP-1 macrophages (2 × 10^5^ cells) in the right flank, respectively.

For GEN therapeutic experiments, SKOV3-derived OCSLCs (1 × 10^5^) and THP-1 macrophages (2 × 10^5^) were mixed with matrigel (1:1), and then 100 μL mixture was injected subcutaneously into each Balb/c-nu mouse. After the xenograft volume achieved about 100mm^3^, the mice were randomly divided into 4 groups, with 4 mice in each group. Group 1 mice were given olive oil by gavage and was considered as control group; Group 2 mice were orally given Genistein dissolved in olive oil (50 mg/kg), once on alternate days, for a total of 10 times; Group 3 mice were intratumorally injected with 20 μL per mouse of adenovirus loaded with pHBad-U6-GFP-shSTAT3 (Hanbio Biotechnology Co. Ltd), once a week, for a total of 3 times; and Group 4 mice were orally given Genistein (50 mg/kg) plus injected the adenovirus expressing STAT3 shRNA. Then, the longest (L) and shortest (W) diameters of the subcutaneous xenografts were measured with a Vernier caliper for volume assessment, according to the following formula: V (transplanted tumor volume, mm^3^) = L × (W)^2^ × 0.5. At the end of the experiment, the mice were euthanized and xenografts were weighed after extraction. Xenograft specimens were fixed in 10% neutral formalin. Tissue sections were submitted to H&E staining, and the histopathological morphology was evaluated by optical microscopy.

### Statistical analysis

Data were analyzed using SPSS 20.0 for Windows (SPSS Inc., Chicago, USA). All the experiments were repeated three times and the data were presented as means±SD. Comparisons between the groups for statistical significance were conducted using a two-tailed Student’s *t*-test. The differences between multiple groups were analyzed by one-way analysis of variance. First, the homogeneity of variance was determined, and all the pairwise comparisons between the groups were analyzed using least significant difference (LSD) method. Tukey’s test was performed in the event of incomplete variance of both the control and the experimental groups. Significance was determined as *p* < 0.05.

The article "Genistein inhibits stemness of SKOV3 cells induced by macrophages co-cultured with ovarian cancer stem-like cells through IL-8/STAT3 axis" was retracted in 2023. Reasons: duplicated images; original data or images not available; unreliable results or conclusions.

## Results

### GEN suppressed M2 polarization of THP-1 macrophages co-cultured with OCSLCs

To determine the effects of GEN on M2 phenotype of THP-1 macrophages co-cultured with OCSLCs, the co-culture system of SKOV3-derived OCSLCs/THP-1 macrophages was used. Figure 1a and b indicated that GEN down-regulated CD163 and p-STAT3 expression of THP-1 macrophage, although the expression of STAT3 showed no significant change. In addition, GEN also decreased the levels of IL-10 (Fig. 1c), increased the levels of IL-12 (Fig. 1c) and nitric oxide (NO) (Fig. 1d) in a dose-dependent manner in Co-CM. Furthermore, we found that the levels of IL-8 in Co-CM were reduced by GEN treatment (Fig. 1e). The similarity findings were observed in OVCAR-3-derived OCSLCs/THP-1 macrophages co-culture (Additional file 1: Figure S1). These results suggested that GEN inhibition of M2 polarization might be involved in decreasing IL-8 secretion and inhibiting STAT3 activation in THP-1 macrophages co-cultured with OCSLCs.

**Fig. 1:** GEN inhibited M2 polarization of THP-1 macrophages co-cultured with OCSLCs. The co-culture of SKOV3-derived OCSLCs with THP-1 macrophages was treated with or without GEN (10, 20, and 40 μM). The levels of CD163 **a** and p-STAT3 **b** protein expression in THP-1 macrophages as well as the contents of IL-10 and IL-12 **c**, NO **d**, and IL-8 **e** in Co-CM were shown.^*^P < 0.05, vs THP-1 macrophages were treated with vehicle (0.1% DMSO). ^*#*^*P < 0.05,* vs THP-1 macrophages were treated with GEN (10.0 μM). These experiments were performed in triplicate

### GEN alleviated stemness of ovarian cancer cells induced by co-CM

To assess the inhibitory effects of GEN on ovarian cancer cell stemness induced by co-culture, the Co-CM from the co-culture system of OCSLCs/THP-1 macrophages treated with or without GEN was obtained. The sphere and colony formation assay revealed that GEN could suppress self-renewal ability (Fig. 2a) and in vitro tumorigenic capabilities (Fig. 2b) in SKOV3 cells induced by Co-CM. Furthermore, compared to vehicle (0.1% DMSO), Co-CM containing GEN from the co-culture system significantly decreased the protein expression levels of the cancer stem cell surface markers CD44, CD133 (Fig. 2c) and the multipotent transcription factors Nanog and OCT4 (Fig. 2d) in SKOV3 cells in a dose-dependent manner. The similarity findings were observed in OVCAR-3 cells induced by Co-CM. (Additional file 2: Figure S2). These results suggested that GEN could also inhibit the stemness of ovarian cancer cells induced by Co-CM.

The article "Genistein inhibits stemness of SKOV3 cells induced by macrophages co-cultured with ovarian cancer stem-like cells through IL-8/STAT3 axis" was retracted in 2023. Reasons: duplicated images; original data or images not available; unreliable results or conclusions.

**Fig. 2:** GEN alleviated stemness of SKOV3 cells induced by Co-CM. SKOV3 cells with Co-CM from the co-culture of SKOV3-derived OCSLCs with THP-1 macrophages and were treated with or without different concentrations of GEN (10, 20, and 40 μM). The sphere and colony formation rate (**a** and **b**, scale bar, 100 μm) and expression levels of CD133 and CD44 (**c**) as well as Nanog and Oct4 (**d**) in SKOV3 cells were shown.*P < 0.05, vs SKOV3 cells induced by co-culture were treated with vehicle (0.1% DMSO). ^*#*^*P < 0.05*, vs SKOV3 cells induced by co-culture treated with GEN (10.0 μM). These experiments were performed in triplicate

### Effects of depletion or addition of IL-8 combined with GEN on M2 polarization of THP-1 macrophages induced by co-culture

Given that the GEN inhibits macrophage M2 polarization co-cultured with OCSLCs and this might be involved in regulating IL-8 secretion, THP-1 macrophages treated with depletion or addition of IL-8 Co-CM in the presence or absence of GEN was prepared. We found that depletion of IL-8 and GEN together suppressed CD163 and p-STAT3 expression (Fig. 3a and b), but not STAT3 expression in THP-1 macrophages, and reduced IL-10 (Fig. 3c) as well as increased IL-12 (Fig. 3c) and NO (Fig. 3d) in the conditioned medium obtained from THP-1 macrophages treated with IL-8 depletion of Co-CM.

**Fig. 3:** Effects of depletion or addition of IL-8 combined with GEN on M2 polarization of THP-1 macrophages induced by co-culture. THP-1 macrophages were treated by depletion or addition of IL-8 Co-CM in the presence or absence of GEN. The levels of CD163 (**a**) and p-STAT3 (**b**) expression in THP-1 macrophages as well as the contents of IL-10 and IL-12 (**c**), NO (**d**) and in Co-CM induced by co-culture in depletion of IL-8 and GEN alone or combination were shown. The levels of CD163 (**e**) and p-STAT3 (**f**) expressions in THP-1 macrophages as well as the contents of IL-10 and IL-12 (**g**), NO (**h**) in Co-CM induced by co-culture by adding IL-8 and GEN alone or combination were shown. *P < 0.05, vs THP-1 macrophages treated with Co-CM. ^*#*^*P < 0.05,* vs THP-1 macrophages treated with conditioned medium obtained from GEN (10.0 μM) treatment. These experiments were performed in triplicate

In contrast, addition of IL-8 significantly abolished the inhibitory effects of GEN on CD163 and p-STAT3 expression of THP-1 macrophages (Fig. 3e and f). ELISA analyses revealed the addition of IL-8 addition exhibited antagonistic activity against GEN on IL-10 and IL-12 secretion (Fig. 3g) as well as NO (Fig. 3h) in the conditioned medium obtained from THP-1 macrophages treated by IL-8 addition to Co-CM. Together, these findings demonstrated that the inhibitory effect of GEN on M2 polarization of THP-1 macrophages required inhibition of IL-8 secretion caused by co-culture.

The article "Genistein inhibits stemness of SKOV3 cells induced by macrophages co-cultured with ovarian cancer stem-like cells through IL-8/STAT3 axis" was retracted in 2023. Reasons: duplicated images; original data or images not available; unreliable results or conclusions.

### Effects of depletion or addition of IL-8 combined with GEN on stemness of SKOV3 cells induced by co-CM

Since GEN could inhibit the secretion of IL-8 through co-culture system, we sought to investigate whether secretion of IL-8 was involved in the effects of GEN on stemness of SKOV3 cells. The results demonstrated that co-treatment of depletion of IL-8 in Co-CM and GEN in co-culture system together attenuated the self-renewal ability (Fig. 4a) and in vitro tumorigenic capabilities (Fig. 4b) in SKOV3 cells. Furthermore, co-treatment significantly decreased the expression levels of CD44 and CD133 in SKOV3 cells (Fig. 4c). Conversely, the addition of IL-8 significantly neutralized GEN decreased the expression levels of CD44 and CD133 in SKOV3 cells induced by Co-CM (Fig. 4d). Addition of IL-8 effectively opposed the GEN attenuated self-renewal ability (Fig. 4e) and in vitro tumorigenic capabilities (Fig. 4f) in SKOV3 cells induced by Co-CM. Together, these findings suggested that the inhibitory effects of GEN on stemness of SKOV3 cells are necessary for the inhibition of IL-8 secretion in co-culture system.

**Fig. 4:** Effects of depletion or addition of IL-8 combined with GEN on stemness of SKOV3 cells induced by Co-CM. SKOV3 cells were treated with conditioned medium from THP-1 macrophages and were treated with depletion or addition of IL-8 Co-CM in the presence or absence of GEN. The sphere and colony formation rate (**a** and **b**, scale bar, 100 μm) and expression of CD133 and CD44 (**c**) in SKOV3 cells induced by Co-CM in depletion of IL-8 and GEN alone or in combination were shown. The sphere and colony formation rate (**d** and **e**, scale bar, 100 μm) as well as expression of CD133 and CD44 (**f**) in SKOV3 cells induced by Co-CM by adding IL-8 and GEN alone or in combination were shown. *P < 0.05, vs SKOV3 cells treated with Co-CM. ^*#*^*P < 0.05*, vs SKOV3 cells treated with the conditioned medium obtained from GEN (10.0 μM) treatment. These experiments were performed at least three times

### Effects of alteration of STAT3 expression combined with GEN on M2 polarization of THP-1 macrophage induced by co-culture

To explore the role of STAT3 activation in GEN inhibition of M2 polarization of THP-1 macrophages, the THP-1 macrophages expressing STAT3 shRNA were initially used in the co-culture system. STAT3 knockdown and GEN treatment alone down-regulated CD163, STAT3 and p-STAT3 expression in THP-1 macrophages, suggesting the suppression of the above by their combined activity (Fig. 5a and b). In addition, STAT3 knockdown and GEN together reduced IL-10 secretion (Fig. 5c) as well as increased IL-12 secretion (Fig. 5c) and NO (Fig. 5d) in Co-CM. Furthermore, we found that the IL-8 levels (Fig. 5e) in Co-CM in response to GEN treatment was further reduced by STAT3 knockdown.

The article "Genistein inhibits stemness of SKOV3 cells induced by macrophages co-cultured with ovarian cancer stem-like cells through IL-8/STAT3 axis" was retracted in 2023. Reasons: duplicated images; original data or images not available; unreliable results or conclusions.

**Fig. 5:** Effects of alterations of STAT3 expression combined with GEN on M2 polarization of THP-1 macrophage induced by co-culture. The co-culture of SKOV3-derived OCSLCs and THP-1 macrophages expressing shSTAT3 were treated with or without GEN. Ad-GFP: the cells transduced with adenovirus expressing GFP. Ad-shSTAT3: the cells transduced with adenovirus expressing shSTAT3. The levels of CD163 (**a**), STAT3 and p-STAT3 (**b**) expression in THP-1 macrophages as well as the contents of IL-10 and IL-12 (**c**), NO (**d**), IL-8 (**e**) in Co-CM induced by co-culture in STAT3 knockdown and GEN alone or in combination were shown. The co-culture of SKOV3-derived OCSLCs and THP-1 macrophages expressing STAT3 were treated with or without GEN. Ad-GFP: The cells transduced with adenovirus expressing GFP. Ad-STAT3: The cells transduced with adenovirus expressing STAT3. The levels of CD163 (**f**), STAT3 and p-STAT3 (**g**) expression in THP-1 macrophages as well as the contents of IL-10 and IL-12 (**h**), NO (**I**), IL-8 (**j**) in Co-CM induced by co-culture in STAT3 knockdown and GEN alone or in combination were shown. *P < 0.05, vs treatment with Ad-GFP. ^*#*^*P < 0.05*, vs co-treatment with Ad-GFP and GEN (10.0 μM). These experiments were performed at least three times

To further identify the role of STAT3 activation in GEN inhibition of M2 polarization of THP-1 macrophages, THP-1 macrophages expressing STAT3 were used in the co-culture system. Our data showed that overexpression of STAT3 attenuated GEN suppressed CD163 and p-STAT3 expression in THP-1 macrophages (Fig. 5f and g). In addition, overexpression of STAT3 abrogated GEN reduced IL-10 secretion (Fig. 5h) as well as increased IL-12 secretion (Fig. 5h) and NO (Fig. 5i) in THP-1 macrophages. In addition, overexpression of STAT3 also abrogated GEN reduced IL-8 levels in Co-CM (Fig. 5j).

To ascertain the role of STAT3 activation in GEN inhibition of M2 polarization of THP-1 macrophage induced by co-culture, THP-1 macrophages expressing STAT3 in those expressing STAT3 shRNA were established. Additional file 3: Figure S3A and B depicted that overexpression of STAT3 attenuated STAT3 shRNA combined with GEN suppressed CD163 and p-STAT3 expression in THP-1 macrophages. In addition, overexpression of STAT3 abrogated co-treatment of STAT3 shRNA and GEN reduced IL-10 secretion (Additional file 3: Figure S3C) as well as increased IL-12 secretion (Additional file 3: Figure S3C) and NO product (Additional file 3: Figure S3D) in THP-1 macrophages. Importantly, overexpression of STAT3 significantly antagonized the inhibitory effects of STAT3 shRNA and GEN co-treatment on IL-8 secretion in Co-CM (Additional file 3: Figure S3E). Collectively, these findings demonstrated that the effects of GEN on M2 polarization of THP-1 macrophages are dependent on the inhibition of STAT3 activation of THP-1 macrophages in the co-culture system.

The article "Genistein inhibits stemness of SKOV3 cells induced by macrophages co-cultured with ovarian cancer stem-like cells through IL-8/STAT3 axis" was retracted in 2023. Reasons: duplicated images; original data or images not available; unreliable results or conclusions.

### Effects of alteration of STAT3 expression combined with GEN on stemness of SKOV3 cells induced by co-CM

To investigate the role of STAT3 activation in GEN inhibition of stemness of SKOV3 cells, Co-CM from the co-culture of OCSLCs with THP-1 macrophages expressing STAT3 shRNA was obtained. The results showed that combination of STAT3 knockdown and GEN together attenuated self-renewal ability (Fig. 6a) and in vitro tumorigenic capabilities (Fig. 6b) in SKOV3 cells induced by Co-CM. As indicated in Fig. 6c, combination of STAT3 knockdown and GEN significantly decreased the expression levels of CD44 and CD133 in SKOV3 cells induced by Co-CM.

**Fig. 6:** Effects of alterations of STAT3 expression combined with GEN on stemness of SKOV3 cells induced by Co-CM. SKOV3 cells were treated with Co-CM from co-culture of SKOV3-derived OCSLCs and THP-1 macrophages expressing shSTAT3 were treated with or without GEN. The sphere and colony formation rate (**a** and **b**, scale bar, 100 μm) and expression of CD133 and CD44 (**c**) in SKOV3 cells induced by Co-CM in STAT3 knockdown and GEN alone or in combination were shown. The co-culture of SKOV3-derived OCSLCs and THP-1 macrophages expressing STAT3 were treated with or without GEN. Ad-GFP: The cells transduced with adenovirus expressing GFP. Ad-STAT3: The cells transduced with adenovirus expressing STAT3. The sphere and colony formation rate (**d** and **e**, scale bar, 100 μm) as well as the expression of CD133 and CD44 (**f**) in SKOV3 cells induced by Co-CM in overexpression of STAT3 and GEN alone or in combination were shown. *P < 0.05, vs treatment with Ad-GFP. ^*#*^*P < 0.05*, vs co-treatement with Ad-GFP and GEN (10.0 μM). These experiments were performed at least three times

To further examine the role of STAT3 activation in GEN inhibition of stemness of SKOV3 cells, Co-CM from co-culture of OCSLCs with THP-1 macrophages expressing STAT3 was obtained. Figure 6d and e indicated that overexpression of STAT3 reduced GEN, which inhibited the self-renewability and in vitro tumorigenic capabilities in SKOV3 cells induced by Co-CM. Overexpression of STAT3 abrogated GEN, decreasing the expression levels of CD44 and CD133 in SKOV3 cells induced by Co-CM (Fig. 6f).

The article "Genistein inhibits stemness of SKOV3 cells induced by macrophages co-cultured with ovarian cancer stem-like cells through IL-8/STAT3 axis" was retracted in 2023. Reasons: duplicated images; original data or images not available; unreliable results or conclusions.

To corroborate the role of STAT3 activation in GEN inhibition of stemness of SKOV3 cells induced by Co-CM, Co-CM from co-culture of OCSLCs with THP-1 macrophages expressing STAT3 in those expressing STAT3 shRNA THP-1 macrophages was prepared. Overexpression of STAT3 reduced STAT3 shRNA combined with GEN, which inhibited the self-renewal ability (Additional file 4: Figure S4A) and in vitro tumorigenic capabilities (Additional file 4: Figure S4B) in SKOV3 cells induced by Co-CM. As indicated in Additional file 4: Figure S4A, overexpression of STAT3 abrogated STAT3 shRNA combined with GEN decreased the expression levels of CD44 and CD133 in SKOV3 cells induced by co-culture. Collectively, these findings demonstrated that the effects of GEN on stemness of SKOV3 cells are dependent on the inhibition of STAT3 activation of THP-1 macrophages in the co-culture system.

### Overexpression of STAT3 rescued the effects of depletion of IL-8 combined with GEN on M2 polarization of THP-1 macrophages induced by co-culture

To clarify whether IL-8/STAT3 axis was involved in GEN inhibition of M2 polarization of THP-1 macrophages, depletion of IL-8 of Co-CM in THP-1 macrophage expressing STAT3 was treated with or without GEN. Figure 7a and b showed that overexpression of STAT3 attenuated depletion of IL-8 combined with GEN, suppressing the expression of CD163 and p-STAT3 in THP-1 macrophages. In addition, overexpression of STAT3 abrogated the depletion of IL-8 combined with GEN reduced IL-10 secretion (Fig. 7c) as well as increased IL-12 secretion (Fig. 7c) and NO product (Fig. 7d) in Co-CM. In addition, overexpression of STAT3 partly attenuated the depletion of IL-8 combined with GEN decreased IL-8 levels in Co-CM (Fig. 7e). These finding suggested that the effects of GEN on M2 polarization of THP-1 macrophage involved IL-8/STAT3 axis in the co-culture system.

**Fig. 7:** Overexpression of STAT3 rescued the effects of depletion of IL-8 combined with GEN on M2 polarization of THP-1 macrophages induced by co-culture. THP-1 macrophages were treated with IL-8 depletion of Co-CM from SKOV3-derived OCSLCs co-cultured with THP-1 macrophages transduced with adenovirus expressing STAT3 and in the presence or absence of GEN. Ad-STAT3: The cells transduced with adenovirus expressing STAT3. The levels of CD163 (**a**) and p-STAT3 (**b**) expression in THP-1 macrophages as well as the contents of IL-10 and IL-12 (**c**), NO (**d**), and IL-8 (**e**) in Co-CM were shown.*P < 0.05, vs treatment with depletion of IL-8. ^*#*^*P < 0.05*, vs co-treatment with depletion of IL-8 and GEN (10.0 μM). These experiments were performed in triplicate

The article "Genistein inhibits stemness of SKOV3 cells induced by macrophages co-cultured with ovarian cancer stem-like cells through IL-8/STAT3 axis" was retracted in 2023. Reasons: duplicated images; original data or images not available; unreliable results or conclusions.

### Overexpression of STAT3 rescued the effects of depletion of IL-8 combined with GEN on stemness of SKOV3 cells induced by co-CM

To determine the role of IL-8/STAT3 axis in GEN inhibition of stemness of SKOV3 cells induced by Co-CM, depletion of IL-8 of Co-CM in THP-1 macrophages expressing STAT3 with or without GEN treatment was prepared. As indicated in Fig. 8a, overexpression of STAT3 abrogated the depletion of IL-8 combined with GEN decreased the expression levels of CD44 and CD133 in SKOV3 cells induced by Co-CM. Figure 8b and c showed that overexpression of STAT3 reduced the depletion of IL-8 combined with GEN inhibited the self-renewal ability and in vitro tumorigenic capabilities in SKOV3 cells induced by Co-CM. These findings demonstrated that the effects of GEN on stemness of SKOV3 cells required modulation of IL-8/STAT3 axis in the co-culture system.

**Fig. 8:** Overexpression of STAT3 rescued the effects of depletion of IL-8 combined with GEN on stemness of SKOV3 cells induced by Co-CM. SKOV3 cells were treated with IL-8 depleting Co-CM from SKOV3-derived OCSLCs co-cultured with THP-1 macrophages transduced with adenovirus expressing STAT3 and in the presence or absence of GEN. Ad-STAT3: The cells transduced with adenovirus expressing STAT3. The sphere and colony formation rate (**a** and **b**, scale bar, 100 μm) as well as expression of CD133 and CD44 (**c**) in SKOV3 cells induced by Co-CM were shown. *P < 0.05, vs treatment with depletion of IL-8. ^*#*^*P < 0.05*, vs co-treatment with depletion of IL-8 and GEN (10.0 μM). These experiments were performed at least thrice

### Combination of GEN and STAT3 shRNA cooperatively inhibited xenograft growth by co-injection of SKOV3-derived OCSLCandTHP-1 macrophages

The results from the nude mouse xenograft model showed that injection with SKOV3-derived OCSLCs alone and co-injection with THP-1 macrophages could form subcutaneous tumors in 30 days; however, the tumor growth by co-injection with OCSLCs/THP-1 macrophages was significantly accelerated than that of injection with OCSLCs alone (Additional file 5: Figure S5A, B and C). Immunohistochemisty revealed elevated human CD68 antigen, IL-8 and p-STAT3 expressions in the co-injected xenografts, compared to OCSLC injection alone (Additional file 3: Figure S3D). These results suggested that the interaction between OCSLCs and THP-1 macrophages promoted the growth of tumors in nude mice in vivo and may be involved in the activation of IL-8/STAT3 signaling pathway*.*

The article "Genistein inhibits stemness of SKOV3 cells induced by macrophages co-cultured with ovarian cancer stem-like cells through IL-8/STAT3 axis" was retracted in 2023. Reasons: duplicated images; original data or images not available; unreliable results or conclusions.

We also found that GEN plus Ad-STAT3 shRNA reduced the size and weight of xenografts in nude mice co-injected with OCSLCs/THP-1 macrophages (Fig. 9a, b and c). The immunohistochemical staining showed that GEN plus Ad-STAT3 shRNA decreased the expression levels of human CD68, IL-8 and p-STAT3 in tumors of nude mice co-injected with OCSLCs/THP-1 macrophages than OCSLCs alone (Fig. 9d). These results demonstrated that GEN inhibits the growth of tumors co-inoculated with OCSLCs/THP-1 macrophages in nude mice in vivo through blocking IL-8/STAT3 signaling.

**Fig. 9:** Combination of GEN and STAT3 shRNA inhibited xenograft growth by co-injection of SKOV3-derived OCSLCs and THP-1 macrophages. The nude mouse xenograft model using co-injection with OCSLCs/THP-1 macrophages was treated with GEN (50 mg/kg) and Ad-shSTAT3 alone or in combination. The size (**a**) volume (**b**), weight (**c**), histological examination (HE staining) and the expression of CD68, IL-8 and p-STAT3 (immunohistochemical staining) (**d**) of xenografts were shown (scale bar, 100 μm). *P < 0.05, vs the model control group; ^*#*^*P < 0.05*, vs treated with GEN (50 mg/kg) or Ad-shSTAT3 alone (means±SD, *n* = 4)

## Discussion

The present study showed that GEN reduced the levels of IL-8 in Co-CM from OCSLCs co-cultured with THP-1 macrophages and inhibited the expression of CD163 and p-STAT3 in THP-1 macrophages, indicating that GEN can reverse M2 polarization of THP-1 macrophages. Moreover, GEN suppressed the sphere and colony formation capabilities and significantly decreased the protein expressions of CD44 and CD133 in ovarian cancer cells induced by Co-CM. These results proved that GEN disrupts the interaction of OCSLCs and TAM, inhibits stemness of ovarian cancer cells induced by co-culture. Therefore, the present study strongly supported the notion that interaction of OCSLCs and TAM contributed to carcinogenicity and progression in human ovarian cancer through elevated IL-8 levels in the microenvironment and activated oncogenic transcription factor STAT3 in THP-1 macrophages co-cultured OCSLCs. This regulation may likely involve the effects of GEN on the prevention and therapy of inflammation-associated cancers, including ovarian cancer.

In addition, activation of IL-8 signal transduction provided tumor cells with chemotherapeutic resistance [28, 29]. IL-8 activates several intracellular signaling pathways in downstream of G-protein-coupled receptor (GPCR) such as CXCR1 and CXCR2 on two kinds of cell surface. The expression of IL-8 and/or its receptors in tumor cells, endothelial cells, infiltrating neutrophils and TAMs has been significantly increased [30, 31]. Nonetheless, the genetic cells were still not decided, and we herein revealed increased IL-8 secretion in Co-CM and similarly its IL-8 levels in SKOV3-derived OCSLCs with THP-1 macrophages co-injected xenografts. In addition, we also demonstrated that alterations of IL-8 concentrations in Co-CM significantly affected M2 polarization of THP-1 macrophage and stemness of SKOV3 cells. Therefore, inhibition of IL-8 signal transduction may be an important therapeutic intervention for targeting tumor microenvironment.

The article "Genistein inhibits stemness of SKOV3 cells induced by macrophages co-cultured with ovarian cancer stem-like cells through IL-8/STAT3 axis" was retracted in 2023. Reasons: duplicated images; original data or images not available; unreliable results or conclusions.

Studies have shown that IL-8 triggers activation of STAT3 signal transduction, which was associated with inflammation, production of reactive oxygen species, tumorigenicity and drug resistance of ovarian epithelial cancer [32–34]. In the present study, we found that knockdown or overexpression of STAT3 in THP-1 macrophages in co-culture system significantly changed the functions that promoted M2 polarization of THP-1 macrophages and stemness of SKOV3 cells induced by co-culture. Furthermore, alteration of STAT3 gene in THP-1 macrophages could change the levels of IL-8 of Co-CM. Given that the STAT3 activation of either CSLCs or TAMs was regulated by varied factors, investigation of STAT3 activation in response to cytokines, chemotactic factors, and other signaling molecules stimulation in tumor microenvironment is conceivable.

Study by Green et al. showed that GEN analogs N-t-boc-Daidzein is used as a new compound for inducing ovarian CSC apoptosis [35]. Our previous studies confirmed that a novel synthetic GEN analogue 7-difluoromethoxyl-5,4′-di-n-octylgenistein (DFOG) effectively inhibited the self-renewal ability of SKOV3-derived OCSLCs [9, 36]. In the current study, we initially provided the evidence that GEN effectively inhibited M2 polarization of THP-1 macrophages and stemness of SKOV3 cells induced by co-culture. Mechanistically, inhibition of M2 polarization of THP-1 macrophages and stemness of SKOV3 cells might be involved in the modulation of secretion of IL-8 in Co-CM and STAT3 activation in THP-1 macrophages in SKOV3-derived OCSLCs and THP-1 macrophage co-culture system. Since IL-8 triggers the activation of STAT3, it is involved in the interaction of tumor microenvironment and CSCs, and can effectively promote the characteristics of CSCs [37, 38]. It is likely that GEN may exert chemoprevention efficacy in several inflammation-associated cancers, not only in ovarian cancer.

Our recent study showed that co-culture of OCSLCs with macrophages induced ovarian cancer cells stemness via IL-8/STAT3 signaling in vitro [15]. Notably, the results observed in the present study proved that the growth velocity of xenografts from co-injection of SKOV3-derived OCSLCs/THP-1 macrophages in nude mice was faster than that of the injection of SKOV3-derived OCSLC alone in vivo*.* More importantly, we demonstrated that co-administration of GEN by gavage and Ad-STAT3 shRNA by intratumoral injection significantly reduced the growth of xenografts by co-injection with OCSLCs/THP-1 macrophages. Therefore, combination of GEN and other STAT3 inhibitors should be a promising and useful therapeutic schedule against inflammation-associated ovarian cancers.

The article "Genistein inhibits stemness of SKOV3 cells induced by macrophages co-cultured with ovarian cancer stem-like cells through IL-8/STAT3 axis" was retracted in 2023. Reasons: duplicated images; original data or images not available; unreliable results or conclusions.

Increasing evidence has revealed the major contribution of TAM in the regulation of stemness of CSLCs through different networks of cytokines, chemokines and growth factors. In these processes, TAM interact with and promote stemness of CSLCs via releasing of milk-fat globule-epidermal growth factor–VIII (MFG-E8) and IL-6 through coordinated activation of the STAT3 and sonic hedgehog pathways [39]. Interestingly, CSLCs are the major subpopulation driving the production of MFG-E8 and IL-6 from macrophages, suggesting that mediators specifically regulated by CSLCs confer macrophages with the ability to promote the generation of tumorigenic factors such as MFG-E8 and IL-6. In return, expansion of CSLC pool lead to stemness maintenance, and immune modulation within tumor microenvironments [40, 41]. In the previous and current studies, we showed the interplay between OCSLCs and TAM accelerates tumor progression through IL-8/STAT3 autocrine positive-feedback mechanisms [15]. Our data provide insight to the molecular interplay between CSLCs and TAMs for inflammation-related human ovarian cancers.

## Conclusions

In conclusion, our study clearly demonstrated that GEN disrupts the interaction between OCSLCs and THP-1 macrophages via blocking IL-8/STAT3 signal axis, reverses M2 polarization of THP-1 macrophages, and inhibits the stemness of SKOV3 cells in transwell co-culture system and co-injection of OCSLC/THP-1 macrophages in nude mice. Although IL-8 is raised from the origin, the potential of the combination of GEN and other STAT3 inhibitors for anticancer activities in inflammation-associated ovarian cancer animal models requires further investigation. Our findings that GEN can inhibit the increased M2 polarization of THP-1 macrophages and stemness of ovarian cancer cells by co-culture of macrophages and OCSLCs through disrupting IL-8/STAT3 signaling axis should be underlined. This in turn assisted GEN to be as a potential chemotherapeutic agent in human inflammation-associated ovarian cancer.

## Additional files

Additional file 1: **Figure S1.** GEN inhibited M2 polarization of THP-1 macrophages co-cultured with OCSLCs. The co-culture of OVCAR-3-derived OCSLCs with THP-1 macrophages was treated with or without GEN (10, 20, and 40 μM). The levels of CD163 (A) and p-STAT3 (B) protein expression in THP-1 macrophages as well as the contents of IL-10 and IL-12 (C), NO (D), and IL-8 (E) in Co-CM were shown.^*^P < 0.05, vs THP-1 macrophages were treated with vehicle (0.1% DMSO). ^*#*^*P < 0.05,* vs THP-1 macrophages were treated with GEN (10.0 μM). These experiments were performed in triplicate. (TIF 32227 kb)

Additional file 2: **Figure S2.** GEN alleviated stemness of SKOV3 cells induced by Co-CM. OVCAR-3 cells treated with Co-CM from the co-culture of OVCAR-3-derived OCSLCs with THP-1 macrophages and were treated with or without different concentrations of GEN (10, 20, and 40 μM). The sphere and colony formation rate (A and B, scale bar, 100 μm) and expression levels of CD133 and CD44 (C) as well as Nanog and Oct4 (D) in OVCAR-3 cells were shown.*P < 0.05, vs OVCAR-3 cells induced by co-culture were treated with vehicle (0.1% DMSO). ^*#*^*P < 0.05*, vs OVCAR-3 cells induced by co-culture treated with GEN (10.0 μM). These experiments were performed in triplicate. (TIF 24203 kb)

Additional file 3: **Figure S3.** Overexpression of STAT3 reversed the co-treatment of STAT3 shRNA and GEN on M2 phenotype of THP-1 macrophages induced by co-culture of THP-1 macrophages expressing Ad-shSTAT3 were transduced with Ad-STAT3 and co-cultured with SKOV3-derived OCSLCs. Ad-shSTAT3: The cells transduced with adenovirus expressing shSTAT3. Ad-STAT3: The cells transduced with adenovirus expressing STAT3. The levels of CD163 (A) and p-STAT3 (B) expression in THP-1 macrophages as well as the contents of IL-10 and IL-12 (C), NO (D), IL-8 (E) in Co-CM were shown. ^*^P < 0.05, vs treatment with Ad-shSTAT3. ^*#*^*P < 0.05*, vs co-treatment with Ad-shSTAT3 and GEN(10.0 μM). These experiments were performed in triplicate. (TIF 33896 kb)

Additional file 4: **Figure S4.** Overexpression of STAT3 reversed the co-treatment of STAT3 shRNA and GEN on stemness of SKOV3 cells induced by Co-CM. THP-1 macrophages expressing Ad-shSTAT3 were transduced with Ad-STAT3 and co-cultured with SKOV3-derived OCSLCs. Ad-shSTAT3: The cells transduced with adenovirus expressing shSTAT3. Ad-STAT3: The cells transduced with adenovirus expressing STAT3. The sphere and colony formation rate (A and B, scale bar, 100 μm) and expression of CD133 and CD44 (C) in SKOV3 cells were induced by co-culture. *P < 0.05, vs treatment with Ad-shSTAT3. ^*#*^*P < 0.05*, vs co-treatment with Ad-shSTAT3 and genistein (10.0 μM). These experiments were performed at least thrice. (TIF 19091 kb)

Additional file 5: **Figure S5.** Co-injection with OCSLC/THP-1 macrophages promoted xenograft growth in nude mice. The xenografts in nude mice were originated from injection with OCSLCs alone or co-injection with OCSLCs/THP-1 macrophages. The size (A), volume (B), weight (C), the histological examination (HE staining) and the expression of CD68, IL-8 and p-STAT3 (immunohistochemical staining) (D) in xenograft tissue were shown (scale bar, 100 μm). ^*^P < 0.05, vs injection with OCSLC alone. (TIF 38543 kb)

The article "Genistein inhibits stemness of SKOV3 cells induced by macrophages co-cultured with ovarian cancer stem-like cells through IL-8/STAT3 axis" was retracted in 2023. Reasons: duplicated images; original data or images not available; unreliable results or conclusions.

## Abbreviations

CSCs: Cancer stem cells
CSLCs: Cancer stem-like cells
DMEM: Dulbecco’s modified Eagle’s medium
FBS: Fetal bovine serum
GEN: Genistein
IL-8: Interleukin-8
L: Longest
LSD: Least significant difference
OCSLCs: Ovarian cancer stem-like cells
SDS-PAGE: Sodium dodecyl sulfate-polyacrylamide gel electrophoresis
STAT3: Signal transducer and activator of transcription 3
TAMs: Tumor associated macrophages
W: Shortest
